# A Combined Approach for Multi-Label Text Data Classification

**DOI:** 10.1155/2022/3369703

**Published:** 2022-06-22

**Authors:** Rokas Štrimaitis, Pavel Stefanovič, Simona Ramanauskaitė, Asta Slotkienė

**Affiliations:** ^1^Department of Information Systems, Vilnius Gediminas Technical University, Saulėtekio Al. 11, LT-10223 Vilnius, Lithuania; ^2^Department of Information Technology, Vilnius Gediminas Technical University, Saulėtekio Al. 11, LT-10223 Vilnius, Lithuania

## Abstract

Automated data analysis solutions are very dependent on data and its quality. The possibility of assigning more than one class to the same data item is one of the specificities that need to be taken into account. There are no solutions, dedicated to Lithuanian text data classification that helps to assign more than one class to data item. In this paper, a new combined approach has been proposed for multilabel text data classification for text analysis. The main aim of the proposed approach is to improve the accuracy of traditional classification algorithms by incorporating the results obtained using similarity measures. The experimental investigation has been performed using the financial news multilabel text data in the Lithuanian language. Data have been collected from four public websites and classified by experts into ten classes manually, where each of the data items has no more than two classes. The results of five commonly used algorithms have been compared for dataset classification: the support vector machine, multinomial naive Bayes, k-nearest neighbours, decision trees, linear and discriminant analysis. In addition, two similarity measures have been compared: the cosine distance and the dice coefficient. Research has shown that the best results have been obtained using the cosine similarity distance and the multinomial naive Bayes classifier. The proposed approach combines the results of these two methods. Research on different cases of the proposed approach indicated the peculiarities of its application. At the same time, the combined approach allowed us to obtain a statistically significant increase in global accuracy.

## 1. Introduction

The amount of unstructured data is increasing at a high rate, and research focusing on such data analysis has evolved. There are various types of unstructured data, such as images, text data, and sounds. The analysis of such data usually leads to uncertainties. First, researchers need to find out the best way to prepare and preprocess data, and later, to choose the best method or model that helps to solve the specific task. There are many different tasks where text analysis is used. Text analysis is commonly applied in text data clustering, classification, sentiment analysis, semantic analysis. For example, text data classification can be applied in the field of security to create spam filters [1] or to prevent cyber-attacks [2], where traditional machine learning algorithms can usually be used [3] such as decision trees, naive Bayes, and support vector machine. There are more fields where text data analysis can be applied: sentiment analysis [4], where the main aim is to detect possible sentiment (positive, negative, neutral) of the text [5]; plagiarism detection to determine the level of similarity of texts, according to the various parts of the text [6]; insurance fraud detection in various areas [7]; and social media data analysis to discover unexpected knowledge that can be used in data mining processes [8]. The most complicated field is the semantic analysis of text, where deep learning algorithms [9] such as long short-term memory, convolutional neural networks, and even the newest methods transformers [10] are used. The main problem in the field of semantic analysis is that one needs not only to classify or cluster the text data, but also the context of the text data taken into account before one or another decision is made.

In most cases of text data classification tasks, the multiclass data is analyzed, where the data items are assigned to only one class from all possible data classes. In this paper, the multilabel text data are analyzed, i.e., the text data items can be assigned to more than one class at once. When the text data are analyzed, it is hard to state unambiguously that data items should be assigned just to one class, especially when the length of the text is high, in such a way the multilabel text data appear. For example, in one part of the text, the text data items can belong to one class and, in another part, to a different class. Therefore, even for experts, it is hard to say which class is more important and which must be chosen. Sometimes, the main class of the text data is considered to be the most frequent word in a text or simply the context of the text.

In this investigation, the multilabel text data collected from four financial news websites in Lithuania have been experimentally analyzed [11]. Each data item is assigned to one or two classes at the same time. There are 10 classes in total. The data collected will be used in the framework of the scientific project to train a model that will be able to predict possible classes of new data. Usually, in the field of text mining, various tasks are performed in which text data are classified, clustered, or searching for similarity between texts. In the case of multilabel text data, there are not many methods to classify such kind of data. Therefore, primary research has been carried out to find out how to improve this type of data classification results using well-known methods of clustering and text similarity. The proposed approach uses the method suggested by other research when binary classifiers are created for each class, but, in addition, the similarity distance is included to improve the overall classification results.

The novelty of the proposed approach gives the possibility of improving the overall classification results by combining commonly used classification algorithms and similarity distance. The proposed approach uses the automatic keyword extraction of each class, or experts can prepare keywords manually. In the case of automatic extraction, the researcher does not have to care about the context of each class, which makes the proposed approach independent of the subjectivity of the person. Furthermore, this research used the multilabel text data adjustment model proposed by Kurasova and Stefanovič [12], which allows improving the quality of the data, as a result, it helps to achieve a higher accuracy of the classification of multilabel text data. The results of the experimental investigation have shown that the combination of classification and similarity measures can be useful and could help other researchers solve such types of classification problem. The experimental investigation has been made using just one multilabel text data set, but the primary research using other languages text shows that the language which has been analyzed does not affect the results of the proposed approach. The only difference is that the data preprocessing has to be modified according to the language of the analyzed text. The results of the proposed approach are promising.

The structure of this paper is as follows. In Section 2, the related works are reviewed. The methods used in the proposed approach are described in Section 3. In addition, in Section 3, the descriptive statistics of the analyzed multilabel text data are presented. Evaluation measures and an experimental investigation of the proposed approach are given in Section 4.  Section 5 concludes the paper.

## 2. Related Works

One of the main tasks of natural language processing is to extract context from text. This can almost always be turned into a text data classification task. The analysis of related works has shown that usually the classification tasks can be defined in four cases: (1) We have a set of texts and we want to assign one label to each of the text data, then the single-label classification task is solved; (2) One of the two labels must be assigned to the text data, for example, whether the text data is positive or negative, then the binary classification task is solved; (3) A multiclass classification task is solved when one of several labels must be assigned to the text data; (4) Usually, in real-life tasks, each text data can have a set of labels, e.g., the book can be described by both horror and detective labels/genres, so in this case, the multilabel classification problem is solved.

When the labels do not correlate, problem transformation algorithms are applied. In the simplest case, the binary relevance algorithm is used; the multilabel classification task is decomposed into a set of binary classification tasks. Unfortunately, labels often indicate dependencies. To address such challenges, Montañes [13] proposed a dependent binary relevance (DBR) model that combines chaining and stacking techniques. The model uses one classifier to produce estimations that mimic true labels, thus detecting label dependencies, and another classifier to predict labels using estimations from the first classifier. The model was tested on 11 different data including text data and compared with the baseline BR, stacking classifier chains, and nested stacking. The results showed that the DBR model was able to achieve better results with the F1, Jaccard Index, and Subset 0/1 loss evaluation metrics, but not the Hamming loss, as the model suffered from mistakes in label estimations during a test phase.

In 2017, Oscar Quispe [14] tried to extract context from several different data that also have financial categories. An attempt was made to classify texts using latent semantic indexing for text representation, a convolutional neural network (CNN) for feature extraction, and a traditional multilayer perceptron for a classifier. In LSI, a singular-value decomposition was used and eight layers-6 convolution layers and 2 fully connected layers were used to construct the CNN model. The rectified linear unit activation function was used in each convolution operation, and the Temporal maximum pooling function was used in pooling operations. Experiments have shown that the proposed solution achieved better results than character-level CNN, bag-of-words, and word2vec if the data documents have more than 1024 characters.

Huang et al. [15] presented a paper proposing the LLSF-DL method to determine label-specific features and class-dependent labels and thus improve multilabel classification algorithms. In the case of label correlation, the author proposes using a high-order label strategy and the model label correlations in a sparse stacking way to reduce error propagation and unnecessary dependent relationships. The method was compared with baseline binary relevance (BR), ensemble classifier chains (ECC), dependent binary relevance (DBR), LIFT, Lasso, GFLasso algorithms, and with LLSF applied to BR, ECC, and LIFT algorithms using ten multilabel benchmark text data. The results showed that LLSF-DL was able to achieve better accuracy, F1, macro F1, and micro F1 than other comparing algorithms, but worse Hamming loss, except for the DBR.

The popularity of transformer's usage to extract context from text increases. Liang et al. [16] proposed a neural hierarchical multilabel text data classification model (F-HMTC) to detect financial events in news documents. The model uses bidirectional transformer encoders for document representation. More than 500,000 news documents from Chinese financial websites were collected to test the model. It managed to achieve better results than other text data classification models: F-HMTC reached 0.7102 hierarchical multilabel distance score (HMD-Score), textCNN-0.5945, Fast Text-0.6113, Hierarchical Attention Network (HAN)-0.6276, and Transformer for text data classification-0.6158.

The efficiency of the model is also influenced by the specifics of the Lithuanian language. At the moment, the analysis of Lithuanian language texts is poorly performed. Krilavičius combined the NLP and IR methods to identify the main topics and facts of the news media [17]. Kapočiūtė-Dzikienė et al. [18] tried to assign one of the three classes—positive, negative, or neutral-to comments from news portals and examined how data preparation affects results. In our previous work [19], we also proposed a classifier to extract sentiment from Lithuanian financial articles. There is no well-known research where the multilabel text data in the Lithuanian language has been used in the classification tasks yet. The main reason for that is the specificity of the Lithuanian language. Usually, models that are suitable and prepared for the English language must be newly trained. In addition, the Lithuanian text data preprocessing differs, because the Lithuanian language is structurally more difficult. Therefore, it is important to develop methods that could help improve overall classification results and can be language independent.

## 3. The Combined Approach for Multilabel Text Data Classification

In this paper, a combined approach has been proposed to classify multilabel text data based on a combination of classification algorithms and similarity measures. The main scheme of the proposed approach is shown in Figure 1.

In the first step, the analyzed multilabel text data must be adjusted according to the approach proposed by Kurasova and Stefanovič [12]. In this way, the quality of the data could be improved. The definition of data quality is related to the problem of determining whether labels were incorrectly assigned by researchers or experts in the data labeling process. This step will be explained in detail in Section 3.2. Later, the analyzed text data are preprocessed to avoid the natural resemblance of the text data and to highlight the core of texts. A binary class assignment has been performed for each text data item. Suppose that we have text data (Table 1), where each text data item belongs to no more than two classes, and there are three classes in total.

In this case, using binary class assignment, the data must be transformed into three subsets (depending on the number of the analyzed data class) with two possible classes, ‘Yes' and ‘No'. These subsets are used to train the binary classifiers in the next step. For example, the data item *X*_1_ belongs to the class ‘Finance' and ‘Politics', so after binary class assignment, this data item will be labelled as follows (Table 2): the class ‘Yes' in the subset of ‘Finance'; the class ‘Yes' in the subset of ‘Politics'; and the class ‘No' in the subset of ‘Industry'. In the same way, the data item *X*_2_ will be assigned to the class ‘Yes' in the subsets of ‘Finance' and ‘Industry', and the class ‘No' in the subset of ‘Politics'. The data item *X*_3_ will be assigned to the class ‘Yes' in the subset of ‘Politics', and ‘No' in the subsets of “Finance” and “Industry”.

After the binary classifiers are trained, the classifiers are used to predict the data class of the new text data items, which has not been used in the previous approach. The other step of the proposed approach is to calculate the similarity distance between the new text data and the keywords of each class. There are usually two options to find keywords: (1) The experts of the analyzed text data have to make lists of words that best represent the classes. (2) The use of automatic keyword extraction algorithms, such as latent Dirichlet allocation [20] can be used. Similarity distances are often used in text mining to find similarities between texts, plagiarism detection, etc. In our proposed approach, the similarity distance helps to decide which list of words the new text data item is most similar to, and in such a way the class is assigned. In both ways, classification prediction and similarity distance complement each other, which help to obtain higher accuracy of the proposed approach. More details about the similarity measure used, the classification algorithm, and the evaluation of the combined approach are presented in Subsections 3.2, 3.3, and 3.4, respectively.

### 3.1. Descriptive Statistics of the Data Analyzed and Data Preparation

The experimental investigation has been carried out using multilabel text data of financial news collected from public websites [11]. The data analyzed is a set of texts *X*_1_, *X*_2_,…, *X*_*N*_, where *N*=12484. Each text data item *X*_*p*_ has been assigned to one or two classes. The classes are as follows: ‘Collective', ‘Development', ‘Finance', ‘Industry', ‘Innovation', ‘International', ‘Law enforcement', ‘Pandemic', ‘Politics', and ‘Reliability'. As was mentioned before, first, the text data have to be preprocessed to reject tokens that are not important and could have an influence on the final results of the proposed approach. The text data preprocessing helps to avoid the artificial similarity between text data. The so-called tokenization has to be performed. Tokenization is a way to separate text data into smaller units called tokens. In this research, tokens can be words, characters, punctuation signs, etc. According to the Kurasova and Stefanovič research [21], the chosen filters are as follows: numbers rejected just as separate tokens but left if a number is a part of a token, for example, ‘covid-19'; all tokens changed to the lower case; the punctuation tokens were erased; the stop list (700 common words) of the Lithuanian language has been used; the tokens that have less than 3 characters have not been included; and the stemming algorithm of the Lithuanian language has been used [22].

The distribution of non-preprocessed text data is presented in Figure 2. As we can see, most of the text data (11475 items) have less than 60 tokens, so the length of the analyzed texts is small. In this research, tokens can be words, characters, punctuation signs, etc. There are 978 text data items for which the number of tokens falls to the interval of (59, 114] and the rest of texts (31 items) have more than 114 tokens. The distribution of preprocessed text data shows that in the majority of the texts (11530 items), the number of tokens is less than 39, the 930 text data items fall to the interval of tokens number (38, 74], and just 23 text data items have more than 110 tokens.

The main problem of the multilabel text data is that it is hard to decide which class is primary, or sometimes the same text can be assigned to more classes than it is labelled. For example, we have the text ‘Many needed the help of lawyers due to the financial problems that arose during the pandemic'. Suppose that this text in the example has to be assigned just to the two classes, so in this case, classes could be ‘Pandemic', ‘Finance', or ‘Law enforcement'. It is hard to decide which two classes represent text the best; it is subjective and usually depends on the opinion of the expert who assigned the class manually. For this reason, in our experimental investigation, we used the original multilabel text data and compared the results with the text data, where the class was adjusted using the approach proposed by Stefanovič and Kurasova [12]. The proposed approach allows automatic multilabel text data class adjustment using latent semantic analysis [23] and self-organizing map [24]. The optimal threshold value was selected to be 85%, as recommended by previous research results [12].

Suppose that we have a text data *X*={*X*_1_, *X*_2_,…, *X*_*N*_} and a bag of words has been created from it. The bag of words is a list of words from all analyzed text data, excluding the words that do not satisfy the conditions defined by the various preprocessing filters. Each data item is described by the words obtained after creating the bag-of-words list. According to the frequency of words in the texts, a so-called text matrix is created:

(1) $$\begin{array}{c} \left(\begin{array}{cccc} x_{11} & x_{12} & \ldots & x_{1n}\\ x_{21} & x_{22} & \ldots & x_{2n}\\ \vdots & \vdots & \ddots & \vdots \\ x_{N1} & x_{N2} & \ldots & x_{Nn} \end{array}\right). \end{array}$$

Here, *x*_*pl*_ is the frequency of the *l* th word in *p* th text, *p*=1,…, *N*, *l*=1,…, *n*. *N* is the number of analyzed texts, and *n* is the number of words in the bag of words. Each row of the matrix is text vector *X*_*p*_′ ∈ *R*^*n*^, *p*=1,…, *N*, which represents a numerical expression of the text *X*_*p*_. In the simplest case, the frequency value is equal to how many words appear in the text. Usually, the relative frequency is used. In this case, the number of frequency words in the text is divided from the total appearance of the word overall in the text data. In addition, in the text analysis, the bag of n-grams could be used. *N*-grams is the method when one word is considered as a unigram, two words-bigram, etc. In this case, the same text matrix (1) is formed, only the elements of the matrix represent unigrams, bigrams, or bigrams and unigrams together. The text matrix of bigrams and unigrams will be used to train classification algorithms and find similarities between text vectors.

### 3.2. Classification Algorithms and Their Evaluation

There are many well-known classification algorithms [25] used in text data analysis, such as decision trees, support vector machine, and deep learning algorithms [26] such as long short-term memory, convolutional neural networks, or even transformers. Therefore, primary research has been done to find which algorithm can better predict the classes of analyzed text data. Because deep learning algorithm's preparation of data is more complicated compared to traditional classification algorithms and requires a bigger number of items in the dataset, in our research we choose to analyze these classifiers: the support vector machine (SVM), Naive Bayes, k-nearest neighbours (kNN), decision trees, linear and discriminant analysis. In the case of multilabel text data, the classifiers have been evaluated by calculating the accuracy, i.e., how the original data classes match the predicted classes obtained by the classifiers. In the primary research, the preprocessed original and adjusted text data have been randomly split into two subsets for training (80%) and testing (20%). To train classifiers, the bag of *n*-grams has been used, which consists of unigrams and bigrams. The frequency of *n*-grams is chosen and equal to 3. As mentioned, the proposed approach uses binary classifiers for each class, so in this case, the same classification algorithm has been used to train 10 classifiers, where each of them can predict whether the data item belongs to the class or not (‘Yes' and ‘No' class). After training the model, the test subset is passed on to the binary classifiers, and the two classes with the highest prediction values are considered assigned classes.

The classification of multilabel text data has its peculiarities for accuracy estimation [27]. In this paper, we use the global accuracy, micro, and macro F1 Score. Also, three additional metrics are used: ‘Perfect match'– the original text data class are the same as predicted, sometimes it is named as ‘Exact Match Ratio ‘; ‘Match'– at least one of the original text data class are the same as a predicted class; and ‘Mismatch'– the original text data class do not match any of the predicted class.

In Figure 3, we can see that the lowest perfect match (7.13%) and the match (49.6%) are obtained using the discriminant analysis classifier, in addition to the highest mismatch (50.40%). Similar results are obtained using SVM, naive Bayes, and linear classification algorithms. The lowest mismatch (11.06%) and the highest match (88.94%) are obtained using naive Bayes. The perfect match is slightly larger using kNN, but only 73.72% of the match value. In the case of adjusted text data, all the results obtained for each classifier are slightly higher (1–2%) compared to the results for the original text data (Figure 4).

The experimental investigation showed that the use of the multilabel text data adjustment approach suggested in the research [12] helps to adjust the original text data class and allows the classifiers to increase the accuracy. The smallest mismatch (10.90%) and the highest match (89.10%) are obtained using naive Bayes, and the perfect match is equal to 21.67%. The highest perfect match is obtained by the linear classification algorithm (22.64%). The worst results were obtained using the discriminant analysis classifier. The research of classification algorithms showed that slightly better results are obtained using the naive Bayes algorithm, so in experimental investigation of the suggested approach the naive Bayes classifier will be chosen.

### 3.3. Similarity Measures

In this paper, the class prediction of new text data has been made according to the classifier's prediction and similarity measure results. Previous work showed that the most common measure of similarity used in text analysis is the cosine distance. Other similarity measures, such as the Dice coefficient, overlap, and extended Jaccard coefficient, can also be used in text similarity detection [28]. In this research, we compared two commonly used similarity measures, the cosine and Dice coefficient, to find out which of them can better predict the class in the case of analyzed multilabel text data. For example, the cosine distance and Dice coefficient between two text vectors *X*_*p*_′, *p*=1,…, *N* can be calculated using the following formulas:

(2) $$\begin{array}{c} \cos\left(X_{1}^{\prime },X_{2}^{\prime }\right)=\frac{X_{1}^{\prime }\times X_{2}^{\prime }}{\sqrt{\left|X_{1}^{\prime }\right|}\times \sqrt{\left|X_{2}^{\prime }\right|}}, \end{array}$$

(3) $$\begin{array}{c} \text{dice}\left(X_{1}^{\prime },X_{2}\right)=2\frac{X_{1}^{\prime }\times X_{2}^{\prime }}{\left|X_{1}^{\prime }\right|+\left|X_{2}^{\prime }\right|}. \end{array}$$

As was mentioned at the beginning of this section, the keyword list of each class has to be formed. Suppose that we have the text data presented in Table 3. Instead of text, the bag of words is given. For simplicity, in this example, the preprocessing filters have not been used. The prepared lists of each class, for example, are as follows: ‘Finance'–prices, financial, money; ‘Industry'–industry, manufacturing; ‘Politics'–government, politics, and president. In this example, only the cosine distance has been calculated to understand how the class prediction is performed. The higher the value of the cosine distance, the more similar the text vectors will be.

In the given example, the relative frequency of words is used. The cosine distance between each list and each text data item is calculated in such a way that the new classes are predicted. The highest values indicate the priority of the classes. Instead of automatic keyword extraction, in this research, the lists have been prepared manually.

In cooperation with a company, the main field of accounting and business management software development with more than 30 years of experience, we chose to collect a list of unigrams and bigrams that best represent the class of analyzed text data. Therefore, the sizes for the lists of each class are as follows: Collective (55), Development (37), Finance (90), Industry (48), Innovation (44), International (59), Law enforcement (74), Pandemic (45), Politics (56), and Reliability (47). Each new text data item that is fed to the proposed approach and the formed lists is preprocessed using the same filters as presented in Subsection 3.1. After that, each new text data item is converted to unigrams and bigrams, the relative frequency is calculated, and the text vector of each class has been formed.

Primary experimental investigation has been performed using the same test subset that has been used in classifier evaluation to determine the accuracy of the prediction of similarity measures. As we can see in Figure 5, the perfect match and match using the cosine distance are slightly lower compared to the results of the Dice coefficient in both cases using the original and adjusted text data. For this reason, in further investigation, the Dice coefficient will be used.

### 3.4. Combined Approach

In primary experiments investigation, the global precision for the classification of text data based on similarity measurement reached 86% (standard deviation 0.23), while the classification of text data reached 82% (standard deviation 0.49). However, when comparing the predicted classes for each method, only 18% of the cases matched (both methods assigned the data item to two identical classes). At least one class was identical between the predictions of these two methods in 69% of the cases, and 13% of cases proposed completely different predictions. Between that 13% of fully different predictions, 4% (similarity measure based) and 11% (text data classification based) of cases were predicting the full match to the assigned classes. Such a mismatch between two models leads to the idea of a combined approach.

Our idea for the combined approach is based on multiple features, generated from similarity measures and binary classification values. We generate such features for combined approach implementation.

(i) Normalized values. Although both the similarity and the binary classifier based values should vary in the interval [0; 1], in practical application, these values might not reach the highest values. Therefore, both values are normalized by dividing them from the maximum value reached in the training data (between all classes).
  (4) $$\begin{array}{c} nv_{m,c,i}=\frac{v_{m,c,i}}{\vee_{k=1}^{cn}\vee_{l=1}^{dn}v_{m,k,l}}, \end{array}$$
where *nv*_*m*,*c*,*i*_ is the normalized value for data item *i*, the class *c* value *v*_*m*,*c*,*i*_ in method *m*. The maximum value for normalization is obtained by finding the maximum value in each class *k* out of *cn* classes and each data item *l* in the training data with *dn* data items in total.
(ii) Data item level normalized values. Some data items have very low values for each class and do not reach the maximum possible value for the method. Therefore, the data items level normalization is executed as well.
  (5) $$\begin{array}{c} rnv_{m,c,i}=\left\{\begin{array}{c} \frac{v_{m,c,i}}{\vee_{k=1}^{cn}v_{m,k,i}},\;\overset{cn}{\underset{k=1}{\vee }}v_{m,k,i}\neq 0,\\ v_{m,c,i},\;\overset{cn}{\underset{k=1}{\vee }}v_{m,k,i}=0, \end{array}\right. \end{array}$$
where *rnv*_*m*,*c*,*i*_ is the data item level normalized value for data item *i*, the class *c* value *v*_*m*,*c*,*i*_ in method *m*. The maximum value for data item level normalization is searched in each class *k* out of *cn* classes for the data item *i*.
(ii) Normalized ranking scores. The distribution of scores between different classes might vary a lot. To change the distribution of value intervals, the ranking of the values are used. As well it is normalized to the interval [0; 1].
  (6) $$\begin{array}{c} rv_{m,c,i}=\frac{cn-\text{rank}\left(v_{m,c,i},\left\{v_{m,1,i},v_{m,2,i},\ldots ,v_{m,cn,i}\right\}\right)}{cn}. \end{array}$$
where *rv*_*m*,*c*,*i*_ is the normalized ranking value for data item *i*, class *c* value *v*_*m*,*c*,*i*_ in method *m*. Function rank (*x*, *y*) return the rank of value *x* in set *y*. The *cn* notes a number of classes in the data while the subtraction of ranking is used to get the ranking in reverse order (from smallest value to highest one).
(ii) Discretized scores. Another method to eliminate the variance of value intervals between different classes is value discretization into a binary value. To do so a threshold value is assigned and all values equal or above it is converted to 1, while lower ones–to 0. The threshold allows the reduction of low importance candidates in cases of very similar classes in the data.
  (7) $$\begin{array}{c} dv_{m,c,i}=\left\{\begin{array}{cc} 1, & v_{m,c,i}\geq t_{m},\\ 0, & v_{m,c,i}<t_{m}, \end{array}\right. \end{array}$$

where *dv*_*m*,*c*,*i*_ is the discrete value for data item *i*, class *c* value *v*_*m*,*c*,*i*_ in method *m*. The *t*_*m*_ defines the discretization threshold value for method *m*.

The combined approach incorporates all these features to analyze a data item and calculate the aggregated values *av*_*c*, *i*_ for each data item *i*, class *c*.

(8) $$\begin{array}{c} av_{c,i}=\left(dv_{sm,c,i}+dv_{cm,c,i}\right)\cdot \left(nv_{sm,c,i}+nv_{cm,c,i}+rnv_{sm,c,i}+rnv_{cm,c,i}\right)+rv_{sm,c,i}+rv_{cm,c,i} \end{array}$$

where *nv*_*sm*,*c*,*i*_, *rnv*_*sm*,*c*,*i*_, *rv*_*sm*,*c*,*i*_, and *dv*_*sm*,*c*,*i*_ are normalized value, data item level normalized value, normalized ranking score, and discretized score, respectively, for similarity method (*sm*), class *c*, data item *i*. Accordingly, *nv*_*cm*,*c*,*i*_, *rnv*_*cm*,*c*,*i*_, *rv*_*cm*,*c*,*i*_, and *dv*_*cm*,*c*,*i*_ are the same metrics for binary classifier method (*cm*).

The predicted classes are selected based on the rank or score of the aggregated value–top *R* values are used to present *R* predicted classes or threshold value *T* is set to estimate the most suitable candidates. We use a combined solution, where the class with the highest score is assigned automatically, while the classes with lower values are assigned based on threshold function *tf*().

(9) $$\begin{array}{c} r=\text{rank}\left(av_{c,i},\left\{av_{1,i},av_{2,i},\ldots ,av_{cn,i}\right\}\right),\\ ca_{c,i}=\left\{\begin{array}{cc} 1, & r=1,\\ tf\left(av_{c,i},r\right), & \text{otherwise}, \end{array}\right.\\ tf\left(av_{c,i},r\right)=\left\{\begin{array}{cc} 1, & \frac{av_{c,i}}{\vee_{k=1}^{cn}av_{k,i}}\geq tfv\cap r\leq tfr,\\ 0, & \text{Otherwise,} \end{array}\right. \end{array}$$

where *r* is a rank of aggregated value *av*_*c*, *i*_ within all *cn* classes aggregated values in the data item. *ca*_*c*, *i*_ is a binary value of either class *c* for the data item *i* should be assigned as predicted class or not. The highest rank class is assigned always, otherwise the aggregated value *av*_*c*, *i*_ for class *c*, data item *i* is assigned by the threshold function *tf*(). The function *tf*() takes into account the proportion between aggregated value and the maximum value of each *k* class within all *cn* classes. If the proportion is greater than the specified class assignment threshold value *tfv* and the rank *r* does not exceed the rank threshold value *tfr*, it is assigned to be a predicted class, otherwise, it is not.

The combined approach application general schema is presented in UML Activity diagram notation (see Figure 6). It illustrated that the data item similarity and binary classification result vectors are used to estimate internal vectors. The final classification results are estimated by combining all the internal vectors and selecting the classes, which meet selection requirements.

## 4. Experimental Investigation

### 4.1. Validation Results

Our combined approach has several parameters, threshold values. For this specific multilabel text data, the discretization threshold values *t*_*m*_ for both similarity and binary classifiers value equal 0. This value was selected taking into account the scores for each class in both methods are low: 72% of similarity scores are equal to 0, while 73% of binary classifier scores have values smaller than 0.05. The discretization threshold values are needed when the false positive rate is too high and needs to be reduced; therefore, it is ignored in the analyzed text data.

Another parameter is the class assignment threshold value *tfv*. As this parameter limits the number of predicted classes, we analyze two cases with more details–one is the false positive reduction oriented case (FPC), when *tfv* = 0.7, and other is the false negative reduction oriented case (FNC), when *tfv* = 0.4.

Our used multilabel text data have one or two classes assigned. Therefore, the limit of the assigned classes *tfr* is equal to 4 in all experiments in this paper. As well, all experiments are executed by using 5-fold cross-validation, where the whole text data are divided into 5 portions (data items selected randomly) and 5 times, one of the data portions is used as testing, new data, while the rest four of them are used for training, maximal value estimation. This allows the estimation of result standard deviation, possible value variations.

In total, 8 different cases are analyzed:

- FPCM–combined approach oriented on false positive reduce using original data.
- FPCA–combined approach oriented on false positive reduce using adjusted data.
- FNCM–combined approach oriented on false negative reduce using original data.
- FNCA–combined approach oriented on false negative reduce using adjusted data.
- SM–similarity approach using original data.
- SA–similarity approach using adjusted data.
- CM–binary classifiers approach with original data.
- CA–binary classifiers approach with adjusted data.

The combined approach (both FP and FN cases) demonstrates higher global accuracy and F1 scores compared to similarity measure or binary classifier approaches (see Figure 7).

The global accuracy achieved for the combined approach varies from 87% (standard deviation 0.8) to 90% (standard deviation 1.0) with different data. Meanwhile, the similarity-based approach was able to reach 86% (standard deviation 0.4) of global accuracy, the binary classifier approach-82% (standard deviation 1.3). Analyzing if the result difference was statistically significant, the *P*-value for the global accuracy of the best combined and noncombined approaches was evaluated as <0.0001. The *P*-value for the worst case of the combined approach and the best of the noncombined approach is equal to 0.0305. As *P*-value <0.05 in both cases, it means that the global accuracy difference between combined and noncombined approaches is statistically significant and the usage of the combined approach brings a significant increase to it.

Similar results are inspected for micro and macro F1 score metrics. Meanwhile, the perfect match and match metrics are not as winning in all cases analyzed for the combined approach. For the FP cases, the perfect match values are one of the lowest (similar to the similarity approach). This is mostly related to class assignment threshold value *tfv*, as it reduces the number of predicted classes. For example, the average number of classes assigned to one data item is 1.47 (standard deviation 0.66) in FP cases. Meanwhile, the number of assigned classes for similarity and binary classifier approaches is 1.79 (standard deviation 0.50) and 2.00 (standard deviation 0.02), respectively. The lower number of predicted classes does not allow matching two assigned classes. Therefore, using the same combined approach with the class assignment threshold value *tfv* = 0.7, the average number of predicted classes is 2.06 (standard deviation 0.92), therefore the perfect match percentage reaches the maximum value of 24% (standard deviation 1.4). It is not a statistically significant difference (*P*-value = 0.1290) compared to the binary classifier that achieved a maximum perfect match score of 22% (standard deviation 2.8).

A perfect match close to 20% should be considered as not bad results taking into account the number of possible combinations between the labels. As there are 10 classes and the data have one or two classes assigned, there are 55 possible combinations overall. If the classifier chose randomly between all possible combinations, the probability perfect match would be 1.8%.

The analog impact of the *tfv* class assignment threshold value is inspected for match score. At least one class will be assigned correctly if the number of assigned classes will be higher, i.e., the *tfv* will be small (see Figure 8).

As the limit of predicted classes is set to 4 (*tfr* = 4), the *tfv* value equals to 0 indicates a case where the first four classes with the highest aggregated values will be assigned as predicted. Four predicted classes are more than enough to achieve 99% accuracy for a match, and at least one class will be assigned correctly. By increasing the *tfv* to 1, the match decreases to 77%. This situation is equal to one when only one class is predicted for multilabel classification. The perfect match value decreases to 0 in the case when *tfv* = 1, as one class is not enough to match two classes. However, global accuracy increases by decreasing the number of predicted classes and reaching 90% when only one class is predicted. This is because we ensure a very high true negative rate–8 classes, out of 10 will not be assigned for sure and will fall into true negative. For the same reason, the standard deviation for global accuracy is very stable and does not depend on the *tfv* value.

The FN cases achieve up to 95% (standard deviation 2.5) match due to the increase of candidates–on average, two classes are predicted. The binary classifier approach has the second biggest number of assigned classes (two highest rank classes are selected), therefore the match value is the second as well–reaches up to 90% (standard deviation 1.5). However, for the match metric comparison between the best results of combined and binary classifier results, the *P*-value is equal to 0.0062, therefore, the difference is statistically significant. If the class assignment threshold value *tfv* would be decreased, the match score would also decrease and with *tfv* = 0.4 it achieves only 89% (standard deviation 2.5) only.

As mentioned above, 13% of data items had no classes in common in similarity-based and binary classifier-based class prediction. After applying the combined approach, 9% of them were classified as perfect matches. While at least one class was assigned correctly (match) by 20% of these data items. As well, it is worth mentioning in cases where neither similarity search nor binary classifier approaches were able to predict at least one class correctly, the combined approach was not able to assign at least one class correctly as well. These data items lack similarity to the assigned class and are worth reconsidering class assignment.

The experimental investigation has been performed using one multilabel text data in Lithuanian language. There are not much publicly available multilabel text data to make a deep comparison on how it will be classified using our proposed approach. Primary research has shown that there is no significant influence when the other language texts are analyzed, but needs to take into account that the entire process of data preprocessing must be chosen according to the language of the text. Nevertheless, the results are promising.

### 4.2. Discussion

The experimental investigation has been performed using one Lithuanian multilabel text data, and the usability of the combination of similarity measure and classifiers results has been experimentally proved. It needs to admit that by using one dataset it is difficult to unambiguously prove the effectiveness of the approach, but the results are promising. The same level of experimental investigation using other multilabel text data has not been performed, because public data with similar properties have not been found. Usually, all the data in the various freely accessed databases are of small size or artificially created. Primary research has shown that the proposed approach is not language-independent. The main difference appears in the text preprocessing step, for example, the specific language stop words have to be included; another stemming algorithm must be used; if the text is longer, the frequency of words may be limited. Also, in the proposed approach, the automatic multilabel text adjustment method has been used presented in previous research which helps slightly to improve the overall accuracy results.

If another dataset would be analyzed that has other or more classes, the list of each class keyword should be prepared, which would be used in the similarity measure calculation step manually or using the automatic keyword extraction methods. This step also can be different and influenced by various factors. Each newly proposed approach has its limitations and threats, but the results of the experimental study are promising and will be used in future work on classification tasks.

## 5. Conclusion

Multilabel text data classification is a complex task because the results can be influenced by various factors, for example, language specificity, data preprocessing, algorithms used to classify, etc. In this paper, the proposed approach is based on two methods: a multinomial naive Bayes classifier and a cosine similarity measure. Additionally, the data adjustment approach has been used to improve the quality of the data analyzed. In this experimental investigation, the multilabel text data items are assigned to one or two classes at the same time. The results of the performed experimental investigation indicate that when just a binary classifier is used, about 20% accuracy can be achieved for a perfect match and about 80% accuracy when at least one out of two classes will be assigned correctly. Meanwhile, when similarity measures are used, the classified data items are compared to predefined keywords and achieve similar accuracy for at least one correctly assigned while the perfect match accuracy decreases to about 10%. This illustrates that unsupervised learning-based solutions are not able to achieve a high perfect match, as supervised learning methods, however, can produce a very similar match of at least one class and, at the same time, do not require data for training.

For multilabel text data classification, the priority between false positive and false negative ratio should be defined, as different approaches produce a different number of assigned classes, which consequently affects the preferred accuracy metric. The proposed combined approach for multilabel text data classification is adaptive and can be adjusted to false-positive or false-negative cases. This adds some adaptability and at the same time allows parameter optimization for the desired purpose (decreased falsely assigned or falsely unassigned class ratio). The proposed multilabel text data classification approach allows for balancing between perfect match and match by estimating the suitable parameters. The balance between parameters of the combined approach allows a statistically significant increase in match classification accuracy in comparison to binary classifiers and usage of similarity measures–the matching of at least one class increased by about 10%.

However, the accuracy of the perfect match does not change significantly and is equal to 20%. I need to admit that in future work, the experimental investigation has to be performed using various multilabel text datasets to fully confirm the reliability of the proposed method. The problem is that there are not many publicly available datasets, especially in Lithuanian.

## Figures and Tables

**Figure 1:** A combined approach for multilabel text data classification.

**Figure 2:** Token distribution of non-preprocessed and preprocessed text data.

**Figure 3:** Classifiers' evaluation using the original multilabel text data.

**Figure 4:** Classifiers' evaluation using the adjusted multilabel text data.

**Figure 5:** Evaluation of the predicted text data class using similarity measures.

**Figure 6:** Principle schema of combined approach application for one data item.

**Figure 7:** Evaluation of predicted classes using different cases and metrics.

**Figure 8:** Impact of the *tfv* value on classification metrics.

**Table 1:** Example of multilabel text data.

ID	Class 1	Class 2	Text
*X*_1_	Finance	Politics	Travel prices increased because of the government decision.
*X*_2_	Industry	Finance	The industry is experiencing financial difficulties.
*X*_3_	Politics		New government elections are coming.

**Table 2:** Multilabel text data after binary class assignment.

ID	Binary classes			Text
	Finance	Industry	Politics	
*X*_1_	Yes	No	Yes	Travel prices increased because of the government decision.
*X*_2_	Yes	Yes	No	The industry is experiencing financial difficulties.
*X*_3_	No	No	Yes	New government elections are coming.

**Table 3:** Example of multilabel text data class prediction using the cosine distance.

ID	Classes	Bag of words	Text matrices	Cosine	New classes
*X*_1_	Finance, politics	Money, and, price, day,government	Finance list (FL) $\left(\begin{array}{ccc} 1 & 1 & 1\\ 0.2 & 0 & 0.2\\ 0 & 0 & 0.4\\ 0 & 0 & 0 \end{array}\right)\begin{array}{c} \begin{array}{c} \text{FL}\\ X_{1}^{\prime }\\ X_{2}^{\prime } \end{array}\\ X_{3}^{\prime } \end{array}$	*d*(FL, *X*_1_′)=0.81	Finance, politics
				*d*(IL, *X*_1_′)=0	
				*d*(PL, *X*_1_′)=0.57	

*X*_2_	Industry, finance,	Industry, money, cars, financial, money	Industry list (IL) $\left(\begin{array}{cc} 1 & 1\\ 0 & 0\\ 0.2 & 0\\ 0 & 0 \end{array}\right)\begin{array}{c} \begin{array}{c} \text{IL}\\ X_{1}^{\prime }\\ X_{2}^{\prime } \end{array}\\ X_{3}^{\prime } \end{array}$	*d*(FL, *X*_2_′)=0.57	Industry, finance
				*d*(IL, *X*_2_′)=0.70	
				*d*(PL, *X*_2_′)=0	

*X*_3_	Politics	Government, elections, president	Politics list (PL) $\left(\begin{array}{ccc} 1 & 1 & 1\\ 0.2 & 0 & 0\\ 0 & 0 & 0\\ 0.3 & 0 & 0.3 \end{array}\right)\begin{array}{c} \begin{array}{c} \text{PL}\\ X_{1}^{\prime }\\ X_{2}^{\prime } \end{array}\\ X_{3}^{\prime } \end{array}$	*d*(Fl, *X*_3_′)=0	Politics
				*d*(IL, *X*_3_′)=0	
				*d*(PL, *X*_3_′)=0.81	

## Data Availability

The data used in this paper are available at https://www.kaggle.com/pavelstefanovi/lithuanian-financial-news-dataset-multilabeled.
